RETRACTED

# Effects of Different Anesthetic and Analgesic Methods on Cellular Immune Function and Stress Hormone Levels in Patients Undergoing Esophageal Cancer Surgery

**DOI:** 10.1155/2022/4752609

**Published:** 2022-03-12

**Authors:** Chaojun Hu, Shan Zhang, Qian Chen, Rong Wang

**Affiliations:** ^1^Department of Emergency, The Affiliated Hospital of Southwest Medical University, Luzhou 646000, Sichuan, China; ^2^Department of Neurology, The People's Hospital of Leshan, Leshan 614000, Sichuan, China; ^3^Department of Neurology, The First People's Hospital of Ziyang, Ziyang 641300, Sichuan, China; ^4^Department of Anesthesiology, The Affiliated Hospital of Southwest Medical University, Luzhou 646000, Sichuan, China

## Abstract

The change of perioperative immune function in patients with esophageal cancer is mainly caused by the joint action of surgical trauma and anesthesia. In our study, we aimed to investigate the effects of different anesthetic methods on the changes of T lymphocyte subsets and cytokines in peripheral blood of patients with esophageal cancer surgery. 50 patients with esophageal cancer were divided into the study group and the control group. Among them, the patients in the control group chose intravenous anesthesia and received self-controlled intravenous analgesia after surgery. Patients in the study group chose thoracic epidural anesthesia combined with general anesthesia, undergoing self-controlled epidural analgesia after surgery; serum interleukin-2 (IL-2) and soluble interleukin-2 receptor (sIL-2R) were measured by ELISA. Serum stress hormones GH and sIL-8 were measured by radioimmunoassay. Both groups of patients achieved significant postoperative analgesia, but the VAS score in the study group at the T2–T4 time point was lower than that in the control group. The serum GH concentration in the study group increased at T1 and reached its highest peak at T2, then decreased. The serum IL-8 concentration of the two groups showed a downward trend from T1 to T4. Thoracic epidural anesthesia combined with general anesthesia for postoperative epidural analgesia can relieve the degree of cellular immunosuppression during and after surgery. Moreover, the thoracic epidural block combined with general anesthesia for esophageal cancer surgery and epidural analgesia after surgery for patients are anesthetic and analgesic methods with clinically significant effects. Our research results have a positive effect on the promotion of postoperative rehabilitation in patients with malignant cell tumors.

## 1. Introduction

Immune function is relatively important in tumor recurrence, metastasis, and prognosis in patients with malignant tumors. Patients with malignant tumors have a relatively low immune function, and major surgery, severe trauma, pain, and anesthesia may result in adverse effects on their immune function, causing severe stress response, unstable homeostasis, and metabolic disorders [1–5]. By performing an analgesic method for stable perioperative anesthesia in patients with malignant tumor surgery, it is possible to fundamentally improve the level of immune function of patients and alleviate or inhibit various harmful and irritating emergency reactions that may be caused by the body, which promotes patients with malignant cell tumors having a positive effect on postoperative rehabilitation [6, 7]. The emergency response induced by trauma in anesthetic surgery will gradually reduce the immune function of tumor patients [8–15]. Many reports have shown that surgical stress inhibition is mainly due to T lymphocyte-mediated cellular immunity, which also has a direct impact on the incidence of postoperative infection and tumor metastasis [16, 17]. A good anesthetic method can reduce the perioperative stress response of patients and protect their immune function [17–21]. Because the degree of cellular immunosuppression during the perioperative period is mainly affected by the size and time of surgical trauma of patients, thoracotomy poses a greater impact on the patient's respiratory and circulatory system [22]. Clinical surgery is more concerned with the patient's stress response, especially in patients with esophageal cancer surgery [23–32]. This index has a certain reference value for the measurement of surgical trauma size.

RETRACTED

This study is mainly to measure the perioperative T lymphocyte subsets and related cytokines in patients with esophageal cancer, to measure the levels of stress hormones at different time points to better understand the different analgesic and anesthetic methods for patients' effects of perioperative immune function and changes in stress response, and to explore the appropriate anesthetic and analgesic methods for patients with esophageal cancer.

## 2. Materials and Methods

### 2.1. Patients

The 50 patients who underwent thoracotomy for selective esophageal cancer in our hospital for the past 3 years were selected as subjects. The age ranged from 38 to 64 years old (56.5  ±  2.5) and the ASA was judged to be in grade I and grade II. All patients did not receive any chemotherapy or radiotherapy before surgery, and their liver and kidney function were normal, and no systemic diseases such as immunity, infection, and endocrine occurred. They were randomly divided into a study group and a control group, with 25 patients in each group. Among them, the patients in the control group chose intravenous anesthesia and received self-controlled intravenous analgesia after surgery. Patients in the study group chose thoracic epidural block combined with intravenous general anesthesia and underwent self-controlled epidural analgesia after surgery.

RETRACTED

### 2.2. Anesthetic Method

Prior to surgery, all patients had 0.5 h to receive the intramuscular injection of phenobarbital sodium (0.1 g) and atropine (0.5 mg). After entering the operating room, the multifunction monitor was selected to monitor systolic blood pressure (SBP), diastolic blood pressure (DBP), heart rate (HR), and mean arterial pressure (MAP); intravenous infusion was also required.

The patients in the control group received anesthetic induction, and Midazolam was selected and its dosage was controlled at 0.05 mg/kg, fentanyl 3 *μ*g/kg, and propofol 1 mg/kg. The patient was injected with 5 *μ*g/kg intravenously before the incision, followed by a continuous intravenous infusion of 5 *μ*g.kg^−1^.h^−1^. Patients in the study group underwent a gap epidural puncture through T_4-5_ or T_5-6_ before anesthetic induction. After that, a mixture of lidocaine and ropivacaine was injected (the two concentrations were controlled at 1% and 5%, respectively). The epidural catheter was injected into the 5 ml mixture after 5 min, and the anesthetic plane was maintained between T_2_ and T_9_. The maintenance dose was injected into the epidural catheter with a 5 ml mixture every 1 h, and the general anesthesia induction cannula was performed after the patient's anesthetic plane was stabilized. The method and measurement are the same as for the control group.

### 2.3. Collecting Blood Specimens

Venous blood in patients were drawn before anesthesia (T0), 2 hours after skin incisions (T1), 24h (T3), and 48h (T4) after surgery, and anticoagulation (2 ml) was selected and sent to a flow cytometer for analysis within 24 hours; 4 ml blood samples were selected for centrifugation in a coagulation tube, and cryopreserved, and the stress response index was measured in a unified time.

### 2.4. Determination of Cytokine

Serum interleukin-2 (IL-2) and soluble interleukin-2 receptor (sIL-2R) were measured by ELISA (enzyme-linked immunosorbent assay) at different time points. Firstly, the number of slats required was selected, and the others were sealed in the refrigerator at 4°C. Secondly, blank holes were placed, and to each blank hole standards and specimens with different concentrations were added, which were controlled to 50 *μ*l. In addition to the blank holes, each hole needs to be added with diluted biotinylated antibodies where their measurement was controlled to 50 *μ*l, then mixed and shaken on the microvibrator. To each hole was added 1 drop of stop solution, mixing it at 450 nm and measuring the OD value. The whole step was controlled to be completed within 5 minutes. To judge the OD value of all standard products/samples, the zero-hole OD value needed to be subtracted, and the standard curve was drawn manually. The standard concentration was taken as the abscissa and the OD value was taken as the ordinate. The coordinate points of different standard products were used to find the specific concentration on the standard line by using the OD value of the specimen.

RETRACTED

### 2.5. Measuring Lymphocyte Subsets

The percentage of CD4^+^T lymphocytes and CD8^+^T lymphocytes was determined by flow cytometry direct immunofluorescence labeling technique, and the CD4^+^T/CD8^+^T ratio was calculated. Flow cytometry used the CellQuest program to analyze the results. The whole cell addition step was first prepared for the single cell suspension. Secondly, the single cell suspension 1^*∗*^106/ml 0.1 ml was selected and added to the mouse antihuman monomer clone antibody working solution at a controlled dose of 0.1 ml, with room temperature being 30 min. Furthermore, the detergent was added to the wash, controlling its measurement to PBS 10 ml. In addition, goat anti-mouse FITC-IgG secondary antibody working solution 100 *μ*l was added, controlled in the dark, incubating for 30 min at room temperature. 10 ml of PBS was added, treated centrifugally, and the supernatant was discarded. 0.1 ml of PBS was added before testing it on the machine, and filtered through 500 meshes of one inch length. Finally, it was tested on the machine.

### 2.6. Determination of Stress Response Index

First, the balance method was used to determine the level of serum cortisol (Cor), selecting the polystyrene tube for numbering, adding standard products, 1251-cortisol, samples to be tested, antiserum, and distilled water, according to the determination of specifications. The bath was set at a temperature of 37°C for 45 min, adding the separating agent and mixing them into the refrigerator, controlling the temperature moderately, controlling the rotation speed to 3500 rpm/min-1 centrifugation for 15 min, aspirating the upper washing liquid. The radioactivity count of different test tube sediments was measured to convert serum cortisol concentration at municipal grade.

### 2.7. Other Indicators Test

Serum interleukin (IL-8), serum prolactin (PRL), and serum growth hormone (GH) were determined by the kit balance method. Polystyrene tubes were selected, numbered, sampled, and centrifuged according to the instructions. The entire procedure was the same as previously described.

RETRACTED

### 2.8. Statistical Method

Statistical software SPSS16.0 was selected to statistically process the relevant data and information. The *t*-test was selected for the group comparison, and the one-way ANOVA was selected for comparison between groups. The data *P* < 0.05 indicated that the difference had statistical significance.

## 3. Results

### 3.1. Comparison of Analgesic Effect of Patients

All patients achieved significant postoperative analgesia. However, the VAS scores of the study group at the T2 and T3 time points were lower than those of the control group, and the difference was significant, as shown in Table 1.

### 3.2. Results of Lymphocyte Subsets in Patients

There was no significant difference between CD4^+^% and CD4^+^/CD8^+^ ratios before anesthesia (*P* > 0.05), and CD4^+^% and CD4^+^/CD8^+^ ratios decreased gradually from T1 in both groups. At T2, the patients in the study group decreased to the lowest level (*P* < 0.01). At T3, the patient's index began to rise in the study group, but at this point, the control group's level was the lowest (*P* < 0.05), and the study group returned to the level between anesthesia at T4, as shown in Table 2.

In the comparison between groups, the CD4^+^% of the study group was higher than that of the control group at T1 to T4. The CD4^+^/CD8^+^ ratio of the study group was higher than that of the control group at T3 to T4. The comparison of CD8^+^ between the two groups at different time points had no statistical significance (*P* > 0.05; Figure 1).

### 3.3. Patients Related Cytokine Changes Results

The changes of patient-related cytokines were dramatically different. The IL-2 levels in the two groups were lower at T1. Its decline was the most obvious at T2. The IL-2 levels of the study group were the lowest. The study group began to decline at T3, and the control group decreased to the lowest. The two groups began to recover at T4, and the control group remained below the preanesthetic level. In the comparison between groups, the IL-2 levels of the study group at T3 and T4 were higher than those of the control group. The levels of SIL-2R in the two groups began to increase from T1 to T4. However, compared with T0, there was no significant difference, which had no statistical significance (*P* > 0.05). There was no significant difference between the two groups that had no statistical significance (*P* > 0.05), as shown in Table 2.

### 3.4. Changes in Serum Stress Hormone Concentration

There was a significant change in serum stress hormone index concentration in patients. The serum GH concentration in the control group gradually increased at the T1 time point. It was the highest peak at T2, and then began to decrease. The GH concentration in the study group did not change significantly. The serum GH concentration in the control group from T1 to T4 was lower than that of the study group. The serum IL-8 concentration of the two groups showed a downward trend from T1 to T4. There was no significant difference in the changes of the control group at different time points. The TI-8 levels in the study group from TI to T4 were lower than those before anesthesia. The decrease of serum IL-8 concentration from T1 to T4 was in comparison, and the decrease in the control group was the most obvious. There was no significant difference in serum Cor in patients at T0 and T1 (*P* > 0.05). From T2, serum Cor in patients increased gradually, reaching the highest peak at T3 (*P* < 0.05) and gradually decreased at T4. However, serum concentration remained exceeding the preanesthesia level, and the serum Cor increased in the study group at T2 and T3, but was lower than that in the control group, as shown in the figure.

RETRACTED

The gray bar chart in Figure 2 shows the corresponding values of GH concentration at different time points in the reference group, while the black one shows the corresponding values of GH concentration at different time points in the study group, with the highest peak at T3. In addition to T0, the GH corresponding values of the whole reference group were higher than those of the study group at several other points (ng/ml).

The gray histogram in Figure 3 shows the corresponding values of PRL concentration at different time points in the reference group, while the black histogram shows the corresponding values of PRL concentration at different time points in the study group, with the highest peak at T2. And the PRL corresponding values of the whole reference group were higher than those of the study group except for T0 (ng/ml).

The gray bar chart in Figure 4 shows the corresponding values of IL-8 concentration at different time points in the reference group, while the black bar chart shows the corresponding values of IL-8 concentration at different time points in the study group, with the highest peak of both values being T0. And the corresponding value of IL-8 in the whole reference group was higher than that in the study group except that T0 was lower than that in the study group (ng/ml).

The gray histogram in Figure 5 shows the corresponding values of Cor concentration at different time points in the reference group, while the black histogram shows the corresponding values of Cor concentration at different time points in the study group, with the highest peak at T3. And the Cor corresponding value of the whole reference group was higher than that of the study group (ng/ml).

RETRACTED

## 4. Discussion

Plasma cortisol and catecholamine concentrations are gradually increased, and immune function is directly inhibited [33–39]. Therefore, the purpose of this study is to find an analgesic and anesthetic method that is more suitable for patients with esophageal cancer surgery.

In this study, patients with esophageal cancer surgery underwent total intravenous anesthesia, thoracic epidural block anesthesia combined with intravenous anesthesia, and observed the postoperative cellular immune function of patients. It is not difficult to find that patients with CD8^+^ levels were not in different periods, but CD4^+^, CD4^+^/CD8^+^ levels began to decrease at the T1 time point, and the study group was the lowest at the T2 time period, gradually began to rise, and returned to the preoperative level at T4. The control group began to rise at the T4 time point. However, it was still below the preoperative level. This indicates that the auxiliary thoracic epidural block can alleviate the decrease of peripheral blood cell immune factor levels in patients, and the relevant indicators of the control group are still lower than the preoperative level at 24 h after surgery, and the study group begins to recover, which means that the epidural analgesia has a relatively low effect on cellular immune function. This study also found that cortisol is an immunosuppressive agent that has been highly studied and can downregulate the patient's immune response. Cortisol can inhibit TH1 cells and amplify the effect of TH2 cells, thereby inhibiting the expression of MHC-II by antigen-presenting cells. Macrophage expression of IL-1 and TNF-*α* was inhibited, inducing the inhibition of body cell immunity. It is not difficult to find that epidural anesthesia can inhibit cortisol secretion and reduce inhibition of cellular immunity.

It is not difficult to find that IL-2 and sIL-2R levels are directly related to T lymphocytes when the immune function of patients is observed. sIL-2R is formed as the *α* chain of sIL-2R, and the expression of sIL-2R in tumor patients is increased, making the role of IL-2 blocked, and inducing T lymphocyte differentiation maturity gradually decreased. In this study, it is not difficult to find that the IL-2 level of the study group is relatively stable in different periods with only a small decrease, and it is restored to the preoperative level at the T4 time point. The IL-2R level is relatively stable, and it has no obvious differences in different time periods. In the control group, IL-2 levels were significantly reduced, and its recovery began at the T4 time point, but it still did not reach the standard level. IL-2 R showed a significant increase, but it still did not return to normal at T4. This means that simple intravenous anesthesia has a stronger inhibition against T lymphocytes, and epidural block combined with general anesthesia has a smaller effect on the levels of different cytokines, and the overall cellular immune function is more stable.

RETRACTED

In this study, it was not difficult to find that even patients with PRL, CH, and Cor levels gradually increased, but related indicators in the study group from T1 to T4 were lower than those of the control group, and IL-8 levels exceeded those of the control group. The comparison of patient's serum Cor concentration showed no significant difference between T0 and T1 (*P* > 0.05). From T2, the serum Cor increased gradually, reaching the highest peak at T3 (*P* < 0.05). It gradually decreased at T4, but the serum concentration still exceeded the preanesthesia level. The serum Cor of patients in the study group increased lower than that of the control group. The VAS score from T2 to T4 time point of the study group was lower than that of the control group (*P* < 0.05), which indicated that the epidural analgesia and analgesic effect were significantly better than those of the intravenous anesthesia.

## 5. Conclusion

In summary, by performing perioperative anesthesia with stable analgesia for patients with malignant tumors such as esophageal cancer, it is possible to fundamentally improve the immune function of patients and alleviate or inhibit various harmful and irritating emergency responses that may be caused by the body, which has a positive effect on the promotion of postoperative rehabilitation in patients with malignant cell tumors. However, there are still some limitations to our research. Future research needs to conduct more experiment analysis and achieve more convincing research results.

## Figures and Tables

**Figure 1:** Changes in CD4 and CD8 in lymphocyte subsets of patients by flow cytometry.

**Figure 2:** GH concentration analysis chart of two groups of patients.

**Figure 3:** PRL concentration analysis chart of two groups of patients.

**Figure 4:** Analysis of IL-8 concentration in two groups of patients.

**Figure 5:** Cor concentration analysis chart of two groups of patients.

**Table 1:** VAS score analysis of patients.

Groups	T2	T3	T4
Control group	3.21 ± 0.34	3.16 ± 0.62	2.80 ± 0.37
Research group	1.65 ± 0.27^*∗*^	1.96 ± 0.47^*∗*^	2.02 ± 0.41

The sign (^*∗*^) symbolized the statistically significant difference (*P* < 0.05).

**Table 2:** Results of lymphocyte subsets in patients.

Immune index groups	Groups	T0	T1	T2	T3	T4
CD4^+^%	Control group	35.72 ± 4.51	30.21 ± 6.21	29.87 ± 5.21	23.45 ± 5.12	28.41 ± 5.12
	Research group	35.72 ± 4.51	30.54 ± 5.17	30.54 ± 5.17	32.81 ± 5.71	36.10 ± 5.62

CD8^+^	Control group	28.21 ± 5.14	28.01 ± 5.14	31.92 ± 6.02	32.45 ± 5.17	28.45 ± 6.15
	Research group	29.41 ± 5.34	28.51 ± 5.24	31.36 ± 6.51	32.18 ± 5.41	29.15 ± 5.91

CD4^+^/CD8^+^	Control group	1.36 ± 0.23	1.04 ± 0.15	0.82 ± 0.12	0.71 ± 0.14	1.03 ± 0.15
	Research group	1.21 ± 0.14	1.07 ± 0.14	0.94 ± 0.11	1.01 ± 0.14	1.21 ± 0.14

IL-2	Control group	13.41 ± 2.61	10.54 ± 5.52	7.84 ± 4.11	7.51 ± 3.84	9.32 ± 3.82
	Research group	13.51 ± 2.54	9.26 ± 4.12	8.64 ± 3.42	9.42 ± 3.14	12.12 ± 4.36

sIL-2R	Control group	648.21 ± 61.21	682.21 ± 57.21	701.34 ± 46.12	681.21 ± 42.21	661.1 ± 50.1
	Research group	650.12 ± 62.41	670.63 ± 56.82	694.81 ± 83.72	681.42 ± 49.62	661.6 ± 50.5

Red data indicate a comparison with T0, *P* < 0.05; italics indicates a comparison with the control group, *P* < 0.05.

RETRACTED

## Data Availability

The datasets used and/or analyzed during the current study are available from the corresponding author on reasonable request.
